This article has been retracted.

# Digital Image Restoration Based on Multicontour Batch Scanning

**DOI:** 10.1155/2022/8106516

**Published:** 2022-09-05

**Authors:** Yongsheng Ding, Yunbo Wei, Shuisheng Zhang, Shihang Yu

**Affiliations:** School of Science Qiqihar University, Qiqihar, Heilongjiang 161006, China

## Abstract

In order to explore the problem of digital image restoration, the authors propose a research on digital image restoration based on multicontour batch scanning. This method recommends key technical problems and solutions based on information represented by multicontour batch scans, exploring research in digital image restoration. Research has shown that the research on digital image restoration based on multicontour batch scanning is about 40% more efficient than traditional methods. Aiming at the new application of digital image inpainting, the application of image inpainting in image compression is studied in depth, and the technical principles of image inpainting and image compression are complemented.

## 1. Introduction

Digital image restoration technology is widely used because of its wide application background; it has become a popular research topic in the field of image processing in recent years [1]. In-depth research on digital image inpainting technology is carried out, and targeted improvements are proposed to improve the image inpainting quality, thereby enhancing the practicability of image inpainting [2]. The application of images is ubiquitous, and a large proportion of the information obtained by human beings in daily life comes from the visual system; with the vigorous development of the computer industry and the advent of the information age, the application value of images as a carrier of information is getting higher and higher. For example, the Bureau of Meteorology can study climate change and environmental pollution through satellite aerial images, and astronomers can study the laws of galaxies by observing astronomical images and observing cosmic celestial bodies such as black holes. Doctors in the hospital inspect relevant parts of the body by taking CT and MRI scans, and the public security department uses fingerprints, faces, and other images to identify and extract the basis for solving cases, etc.; the development of more and more technologies requires the use of images; it can be said that the development of modern technology is inseparable from images.

The concept of “image restoration” originally originated from the restoration of ancient paintings and other works of art [3]. Some cultural relics such as calligraphy and painting are damaged to a certain extent due to environmental factors, human factors, and other factors during the preservation process, such as scratches and missing [4]. The initial image restoration is to repair and fill in the damaged parts of the work by specialized experienced art maintainers; the purpose is to restore the damaged image into a complete and clear work as much as possible by means of image restoration, which is the predecessor of image restoration technology. There is undoubtedly a great risk in directly repairing the original precious artwork; some simple negligence and carelessness may lead to unpredictable consequences or even irreversible losses. With the realization and popularization of image digitization, a new restoration idea has emerged, which can scan the original work into digital form and store it in the computer and only need to use the image restoration technology to perform related processing on the scanned digital files. In this way, manipulation of the original work can be avoided, which greatly reduces the risk of repairing the image. In the above-mentioned “correlation processing,” image restoration technology plays a pivotal role; after years of research and development, digital image restoration technology has now developed into an increasingly mature subject.

Due to the advent of the mobile Internet era and the medical information revolution, images and videos have become more and more popular, and image processing has received more and more attention and has developed into a promising discipline [5]. Images will inevitably be damaged in the process of acquisition and transmission, which undoubtedly brings great difficulties to researchers. For different processing purposes, image processing is mainly divided into image enhancement, image restoration, image reconstruction, and image segmentation.

In recent years, the popular wavelet transform has developed very rapidly and has gradually become the frontier and hotspot in the field of image compression [6]. Wavelet transform takes into account the visual characteristics of the human eye while eliminating image redundancy and has a wide range of applications in the field of compression of static images and dynamic images [7]. The image compression of wavelet transform has greater advantages than discrete cosine transform, it has high compression ratio and no block effect, it has strong processing ability for detail noise and can display image data at multiple resolutions, and therefore, the image compression method based on wavelet transform replaces DCT and becomes a main research direction in the field of image compression. The current popular JPEG200O is a new standard for image compression based on wavelet transform, as shown in Figure 1.

## 2. Literature Review

Jiao and Wu said that since images are a direct way for people to obtain information, the processing of images is particularly important [8]. With the development of modern science and technology, image processing technology has been widely used. Choi et al. said that in the field of medical research, radiography and micrographs have been used to diagnose diseases for a long time [9]. Jiu and Pustelnik said that at present, computer image processing has become an important processing method for disease diagnosis [10]. Agnes et al. said that the internal conditions of the body that were previously undetectable by general inspection methods can now be obtained by special medical imaging modalities [11]. One of the most representative diagnostic methods is X-ray CT (computed tomography). The development of digital image processing and reconstruction to today's level is mainly due to (1) the development of the computer itself. Early computers were difficult to meet the requirements of real-time processing of massive data in terms of processing speed and storage capacity. With the development of computer hardware and digital technology, the prices of computers, storage devices, and peripheral devices have dropped sharply, and their performance has been significantly improved. Processing that was previously only possible with mainframe computers is now possible with personal computers. (2) The development of mathematics. In particular, the emergence and development of discrete mathematics has laid a theoretical foundation for digital image processing.

Zheng believed that people usually process images in order to obtain high-quality images in order to achieve satisfactory results [12]. For example, removing noise in the image, enhancing or suppressing some parts of the image, or changing the brightness of the image thereby improves the quality of the image. Neilson et al. believe that extracting information or certain features contained in images to facilitate computer analysis is also a factor that people consider image processing, including preprocessing for computer vision [13]. Espriella et al. believe that the last reason is to facilitate the storage of images, so as to complete the encoding and shrinking of images [14]. Digital image processing mainly includes geometric processing, image coding, image enhancement, image restoration, image reconstruction, and image segmentation. Any image processing process can be simply modeled using an input-output system. Unfortunately, most image processing problems are ill-posed inverse problems that do not satisfy uniqueness, existence, or stability. Therefore, how to solve ideal solutions from these underdetermined problems brings great challenges to people. Since the image is disturbed in the process of acquisition, transmission, or storage, the image will be degraded; for example, the image contains noise and is blurred. Therefore, prior knowledge of the degenerate system is used to construct suitable mathematical models to reduce or eliminate the distortion of the observed images, resulting in high-quality images that are easy to observe and study.

The idea of image restoration has a long history, but it is a relatively new topic in the field of image processing to be studied as a technology. Until 2000, the concept of image restoration (image inpainting) was introduced at the International Graphics Annual Conference, a more formal and internationally influential conference, formally proposed by Bertalmio et al. Since then, digital image restoration technology has become a general term for a type of work that uses computer programs to run autonomously, or to restore missing images with a small amount of human-computer interaction. Image restoration is not only a simple image processing problem but also involves many fields such as computer vision, computer graphics, and human visual psychology; there are many influencing factors and various processing methods, and because of its high practical value, it has attracted the research of many scholars; the related technology of digital image restoration has become a relatively popular research topic.

Because digital image restoration technology involves technologies in many fields, various research methods emerge one after another, and the classification of image restoration methods is also different based on different classification standards. According to different inpainting ideas and focus, digital image inpainting can be simply divided into two categories: structure-based inpainting methods and texture-based inpainting methods. Most of the structure-based image inpaintings are processing methods in the form of solving partial differential equations; the main idea is to imitate the skills of manual inpainting and gradually diffuse from the boundary of the missing area to the interior through an iterative method to achieve image filling. In the original repair scheme proposed, iterative repair is performed in sequence from the outside to the inside along the isoilluminance line with a single pixel as the basic unit; the repair process is realized by solving a third-order PDE, which is based on an early classical approach to the structure of the BSCB model. The repair idea and mathematical modeling of the BSCB model are easy to understand and implement, but the repair feature of this repair method is based on pixels, which determines that the repair speed must be very slow, and the repair effect lacks overall beauty and coordination; therefore, the BSCB model is often only used as a reference model for image inpainting.

## 3. Methods

### 3.1. The Process of Adding Blur and Poisson Noise

Typically, blur and Poisson noise are added to the process, where *u* is the real image, *H* is the blurred point spread function (PSF), and Poisson represents the effect of Poisson noise [15, 16]. The formula for this problem is shown in

(1) $$\begin{array}{c} z=\text{Poisson}\left(Hu\right). \end{array}$$

Degradation of acquired signals caused by Poisson noise is a common phenomenon in applications such as biomedical imaging, night vision, and astronomy [17, 18]. Therefore, Poisson noise removal is especially important for further processing such as image classification and recognition. Poisson noise is a type of signal-dependent noise. It is very different from Gaussian noise and does not satisfy the simple additivity principle, so the commonly used Gaussian noise removal algorithms cannot be directly applied to Poisson noise suppression. Specifically, assuming that the observed noise-contaminated image obeys a Poisson distribution, the discrete probability is shown in

(2) $$\begin{array}{c} P\left(f\left|u_{i}\right.\right)=\frac{e^{-u}u^{f}}{f_{i}!}. \end{array}$$

In the subetwork SubNet1, Taylor's formula and convolution operator are successively employed to simulate the generalization of the regular forward transform. More specifically, by introducing a transformation and applying Taylor's formula, it can be obtained as shown in

(3) $$\begin{array}{c} gi=2\sqrt{\frac{fi+3}{8}}. \end{array}$$

The convolutional operator created by “Conv” is usually an integral part of the convolutional neural network architecture. Each convolutional layer is a neuron with learned weights {*w*} and biases {*b*}, as shown in

(4) $$\begin{array}{c} y_{i2,j2,d2}=\text{Conv}{\left(x\right)}_{i2,j2,d2}. \end{array}$$

First, for stability purposes, the equation is generalized using the multiple “Conv” layers and summation operators in SubNet1, i.e., as shown in

(5) $$\begin{array}{c} g\approx \sqrt{\frac{6}{2}}+2\sqrt{\frac{6\varphi f}{3}}, \end{array}$$

(6) $$\begin{array}{c} g\approx \text{Conv}\left(1\right)+\text{Conv}\left(f\right). \end{array}$$

Suppose there is a damaged image *I*, the middle irregular area *Q* is the area to be repaired, *t* is the boundary, and the known area is in it. The repair process is an iterative process that gradually diffuses along the image boundary in a coarse-to-fine and external-to-interior manner, and its iterative equation can be expressed as

(7) $$\begin{array}{c} I^{n+1}\left(i,j\right)=I^{n}\left(i,j\right). \end{array}$$

In the formula, *n* is the number of iterations, *n* + 1 is the current number of iterations, (*i*, *j*) is the pixel coordinates in the two-dimensional image, and Δ*t* is the step size of each iteration, which can usually be set to one constant value. The improvement amount is a key amount in the formula, which is directly related to the diffusion mode of the repair process; its calculation expression is shown in

(8) $$\begin{array}{c} I_{t}^{n}\left(i,j\right)=\bar{\delta L}\left(i.j\right)\bar{N}\left(i,j\right). \end{array}$$

The CDD model is the curvature-driven diffusion model; on the basis of the TV model, the curvature-driven term *s* is introduced into the expression of the diffusion intensity factor; its mathematical expression is shown in

(9) $$\begin{array}{c} s=\nabla \left(\frac{\nabla I}{\left|\nabla I\right|}\right). \end{array}$$

For the convenience of calculation, we can simply take *g*(|*s*|) = |*s*|, so as to obtain the repair expression of the CDD model as shown in

(10) $$\begin{array}{c} -\nabla \left[\frac{g\left(\left|s\right|\right)}{\left|\nabla I\right|}\nabla I\right]+\chi \left(I-I_{0}\right)=0. \end{array}$$

The values in Table 1 show that the three convolutional filters are indeed similar in terms of quantitative metrics [19, 20]. In particular, the network trained with the Gaussian blur kernel is more correlated than the other two blur kernels. Second, the transform layer in the residual subnet contains not only smooth features but also some detailed features similar to noise. That is, the residual block does play a role in non-Gaussian noise removal, as shown in Table 1.

## 4. Results and Analysis

For the convenience of comparison, the repair time and various repair indicators of the above three groups of experiments are listed in a table [21]. The number of repaired pixels of the image to be repaired is directly related to the repair time; the more pixels to be repaired, the longer the repair time is required. The total number of repaired pixels reflects the search range of the sample block, which indirectly affects the repair time; the ratio of repaired pixels to total pixels can also reflect the difficulty of image repairing. The number of sample replications reflects the specific number of block replications in the repairing process; this parameter is determined by the average size of the replicated blocks, which can indirectly reflect texture complexity and structure information of the block to be repaired. The influence of the number of Poisson treatments to the number of sample replications on the repair time is also an important parameter worth referring to [22, 23]. It can be seen from Table 2 that the repair time of the three images to be repaired is in the unit of 100 seconds, which is within the acceptable range, and the proportion of repaired pixels to the total pixels is 3.5%, 6.8%, and 20.0%, different loss ratios represent different inpainting difficulties, and all three groups of images to be inpainted with different ratios have been inpainted, indicating that the proposed inpainting algorithm has good versatility [24, 25]. In the three groups of experiments, the number of Poisson processing accounts for about 20% of the total number of sample replications; it can be verified that Poisson processing indeed repairs only the outermost circle of sample blocks as expected. The algorithm repair indicators are shown in Table 2.

In the field of image restoration, there is currently no reliable and consistent objective evaluation standard for restoration effects; the most widely used in traditional restoration technology researchers is peak signal-to-noise ratio; since the object removal experiment does not have a known image as a comparison benchmark, this index cannot be calculated, so this objective evaluation criterion cannot be applied in the repair experiment in such a situation. This experiment uses a subjective evaluation criterion; that is, the observer evaluates the inpainted image without knowing the inpainted area [26, 27], as shown in Table 3.

As shown in Table 3, the repair method used in the experiment has achieved good results in terms of repair time and repair quality; the traditional Criminisi AIEI model has the shortest repair time; however, it is difficult to guarantee the repair quality for a specific image; the proposed improvement method improves the repair quality to a certain extent, but it increases the time cost significantly; the proposed improvement method can significantly improve the image repair quality without increasing too much repair time, which is an effective improvement scheme.

The discrete cosine transform can play a role in concentrating the data energy of the correlation in the image; after the DCT transform, the image information is concentrated in the upper left corner of the matrix; it represents the low-frequency component of the image, and most of the image information is reflected here. While most of the values in the lower right part are zero or near-zero fractional values, this information represents the high-frequency components of the image. Before performing inverse discrete cosine transform, discarding these coefficient values close to zero has little effect on the picture quality of the reconstructed image but achieves the purpose of expressing the image with less data, thus enabling the compression of image data [28].

After the original image is subjected to discrete cosine transform and some coefficients are discarded, the coefficient matrix is coded, and the compression method adopts relatively simple RLE coding. RLE coding is also known as run-length coding; during image coding, adjacent elements with the same pixel value in a specified direction are defined as a round, and the length of the retention is a continuous run, referred to as a run for short. The main principle of run-length coding is to represent the same value string in the image matrix with a representative value plus the run length, so that the representation length of the matrix data is smaller than the length of the original data, thereby realizing data compression.

The selection of reserved block and discarded block is a key step in image inpainting applied to image compression; if there are too few discarded blocks, it is not conducive to improving the compression ratio; and if there are too many reserved blocks, it is difficult to guarantee the repair effect. Especially if important feature blocks are discarded by mistake, it will cause no repair or obvious repair traces after repair. Therefore, the goal to be achieved in this step is to find the most suitable balance between discarding redundant blocks and retaining important feature blocks. The method adopted is to extract the edge of the compressed image first and then sharpen it; at the same time, the extreme points in the image block are counted; Finally, the pixel on the sharp edge and all the extreme points of the statistics are processed, that is, the expansion processing. Then all the selected blocks can be obtained and then the unselected blocks will be deleted.

The edge of an image generally refers to the position where the gray value of the image changes significantly, the principle of edge detection is usually realized by using the differences in gray, color, and texture characteristics between the object and the background; common detection operators include Prewitt operator, Robert operator, Sobel operator, and Canny operator.

The Canny edge detection operator can process image edges from multiple stages such as filtering, enhancement, and detection, and its gradient is calculated using the derivative of the Gaussian filter. First, smooth the image with a Gaussian filter, then calculate the magnitude and direction of the filtered image gradient, and then apply nonmaximum suppression processing to the gradient value; finally, the double threshold method is used to connect the edges.

Considering that the image matrix is composed of discrete pixels, the above operators all use the difference method to approximate the partial derivatives. The adopted edge detection and sharpening methods are as follows: first, the Sobe1 horizontal edge sharpening filter is used to extract and sharpen the image edge, and then, the Prewitt horizontal edge filter is used to extract and sharpen the image twice. Sharpening twice with different filters can obtain contours that are beneficial to inpainting. The source point of the image is a key point with strong structure, usually such a key point is a mathematical extreme point, and the extreme point includes a maximum point and a minimum point, and such key points are calculated and marked. The image to be repaired can be obtained by expanding the extracted and sharpened contours and the obtained source points by several pixel widths.

Table 4 is a comprehensive comparison of the three groups of experiments; after using the compression scheme of this experiment for compression and redundancy elimination, each can obtain different compression ratios. By vertical comparison, it can be found that the overall compression ratio is related to the encoding and decoding method used in the first compression and the redundancy elimination amount of the second “compression”, and the encoding and decoding processing of the first compression scheme of the three images and the redundancy elimination method in the second “compression” are the same, but since the redundancy of the three images themselves are different, this leads to the difference in the amount of culling, which directly leads to the difference in the compression rate. Horizontal comparison, the choice of the image restoration method after secondary “compression,” has a very important influence on obtaining a complete image; the CDD restoration model can be judged from the objective evaluation index of PSNR (peak signal-to-noise ratio); the AIEI repair model and the repair effect of the repair method used in the experiment show an increasing trend, as shown in Table 4.

Three sets of experiments demonstrate the feasibility of applying image inpainting to image compression; however, since the inpainting mechanism of image inpainting technology uses the correlation of the image itself, therefore, the prerequisite for applying image restoration technology to image compression is that the image content has a certain correlation. If the correlation of the image is large, a relatively large compression ratio can be obtained, but if the image itself is an image with low correlation and complex texture, the compression ratio obtained by this scheme will be correspondingly reduced. For example, the image in experiment 3 is relatively complex due to its relatively complex texture; the obtained compression ratio is lower than that of experiments 1 and 2.

The compression ratio obtained by this scheme is limited, and the highest compression ratio obtained in the three groups of experiments is less than 5 : 1, while the compression ratio that can be achieved by the existing mainstream compression standard JPEG is usually above 10 : 1; the emerging development of JPEG2000 can even achieve more, indicating that the compression ratio obtained by this scheme cannot be compared with special compression standards. As far as the compression ratio is concerned, the application of digital image restoration technology to image compression cannot establish its own advantages, but the significance of this scheme is an attempt to a new compression idea other than traditional compression methods; from this perspective, the scheme of applying image inpainting to image compression enhances the flexibility of image compression techniques. Compared with traditional compression methods such as JPEG, the scheme applying image restoration to image compression has the capability of restoration processing in addition to compression. If the image itself is damaged after compression by JPEG compression, the desired image cannot be recovered due to no follow-up processing mechanism; on the contrary, this scheme can repair the damage caused by the compression itself due to subsequent repair processing; thus, the fault tolerance of compression can be enhanced.

At the same time, the compression ratio that can be obtained by this scheme is also directly related to the restoration capability of the image restoration technology; when the image is fixed, the reason why a higher compression ratio cannot be obtained is because the existing digital image restoration technology has considerable limitations on the restoration ability of compressed images. For the restoration after compression, the restoration algorithm obtains a better restoration effect than the CDD model and the AIEI model. The compression ratios obtained in the three sets of experiments are all the maximum values obtained under the premise that the repair algorithm studied can be repaired; that is, in the case of more discarded blocks, the existing repair algorithms have been difficult to complete the repair task. In theory, with the further development of image restoration technology, under the condition that the new repair technology has more powerful repair ability, a higher compression ratio can be obtained.

Since VST-Net-joint performs better than VST-Net-part, this section only discusses VST-Net-joint. Some variants of the network VST-Net-joint are studied from different aspects, i.e., with/without BN layers in SubNet2, the number of Conv layers in SubNet1 and SubNet3, and the number of channels and filter sizes in the entire network. First, the proposed networks with and without BN layers are compared in SubNet2.  Figure 2 lists the average PSNR and SSIM values on Set11. It can be seen that in the network with BN layers, it can achieve better performance with regard to medium and large peaks. Conversely, in terms of peaks, better performance can be obtained in networks without BN layers. This phenomenon shows that the first stage used for variation stabilization is indeed imprecise, and the noise produced subsequently in the second stage is not exact Gaussian noise. BN layers are great for removing Gaussian noise, not for non-Gaussian noise, as shown in Figure 2.

## 5. Conclusion

Image restoration and reconstruction have always received extensive attention from researchers. Traditional algorithms can achieve satisfactory results to a certain extent, but with the increasing maturity of convolutional neural networks, network learning algorithms have brought more research directions to people. The work mainly focuses on image restoration and reconstruction based on convolutional neural networks; first, the network is simply constructed; after the image deblurring has a certain effect, the network is improved to make it better applicable to Poisson image denoising task. Subsequently, medical CT images were explored.

The application of image restoration is studied, including conventional applications such as restoration of art works, cultural relics, photo text removal, and new applications such as relatively complex video transmission error concealment and virtual scene generation, the application feasibility of image inpainting in the above application fields is expounded, and relevant application examples are made by using the existing image inpainting technology. A “secondary compression” scheme is proposed by extracting and removing information from conventionally compressed images and then repairing the compressed images with restoration technology to obtain complete images for normal use.

## Figures and Tables

**Figure 1:** Compression scheme combining image inpainting and image compression.

**Figure 2:** Average PSNR (dB) and SSIM values with/without BN in SubNet2.

**Table 1:** Correlation values between the first Conv convolutional layers of the training network.

	Conv-kernel-Gaussian	Conv-kernel-average	Conv-kernel-motion
Conv-kernel-Gaussian	1.01	0.89	0.88
Conv-kernel-average	0.81	1.04	0.83
Conv-kernel-motion	0.89	0.83	1.08

**Table 2:** Algorithm repair indicators.

Indicator records/experimental images	Table	Horse	Jumper
Repair time (s)	130.38	197.63	97.28
Repair pixel(s)	3426	6730	12690
Total pixels (pieces)	98304	98304	63448
Sample replication times (times)	134	212	225
Number of Poisson treatments (times)	35	49	40

**Table 3:** Comparison of repair evaluation and repair time.

Experimental image/repair method		Criminisi repair	Regular Poisson processing fix	Repair method used in experiments
Table	Subjective evaluation (score/total score)	7.1/10.0	8.1/10	8.8/10
	Repair time (s)	11903	140.43	130.36
Horse	Subjective evaluation (number of approvals/sample)	6.2/10	6.5/10	8.1/10
	Repair time (s)	188.71	226.03	197.63
Jumper	Subjective evaluation (number of approvals/sample)	5.2/10	7.2/10	8.3/10
	Repair time (s)	90.23	112.81	97.28

**Table 4:** Comparison of compression and repair schemes.

Number of experimental groups	Original image size (KB)	Compressed size (KB)	Compression ratio (%)
Experiment 1	65.12	15.04	23.47
Experiment 2	65.27	14.78	22.92
Experiment 3	88.17	28.37	32.73

## Data Availability

The data used to support the findings of this study are available from the corresponding author upon request.

## References

[1] Gao X. M., Li Y. L., Lu B. L., Xiong Q. X., Li J. F. (2021). Estimation of spad value in waterlogged winter wheat based on characteristic indices of hyperspectral and digital image. *Ying yong sheng tai xue bao = The journal of applied ecology/Zhongguo sheng tai xue xue hui, Zhongguo ke xue yuan Shenyang ying yong sheng tai yan jiu suo zhu ban*.

[2] Sindu B. S., Thirumalaiselvi A., Sasmal S. (2021). Investigations on fracture related properties of strain hardened concrete using digital image correlation and acoustic emission techniques. *European Journal of Environmental and Civil Engineering*.

[3] Khalilzadehtabrizi S., Seifiasl A., Asl M. H. (2021). Measurement of deformation patterns in steel plate shear walls subjected to cyclic loading based on multi-target digital image correlation (MT-DIC). *Structure*.

[4] Haq T. U., Shah T., Siddiqui G. F., Iqbal M. Z., Jamil H. (2021). Improved twofish algorithm: a digital image enciphering application. *Access*.

[5] Jing G., Du Y., You R., Siahkouhi M. (2022). Comparison study of crack propagation in rubberized and conventional prestressed concrete sleepers using digital image correlation. *Proceedings of the Institution of Mechanical Engineers, Part F: Journal of Rail and Rapid Transit*.

[6] Kai Y., Ogawa T., Wang Z., Adachi Y. (2021). Strain distribution analysis of two perpendicular planes in sus310s austenitic stainless steel using digital image correlation. *ISIJ International*.

[7] Ahmed W. M., Verhaeghe T. V., McCullagh A. P. (2021). Maxillary complete-arch implant-supported restoration: a digital scanning and maxillomandibular relationship workflow. *The Journal of Prosthetic Dentistry*.

[8] Jiao J., Wu L. (2020). Image restoration for the mra-based pansharpening method. *Access*.

[9] Choi K., Lim J. S., Kim S. K. (2020). Statnet: statistical image restoration for low-dose CT using deep learning. *IEEE Journal of Selected Topics in Signal Processing*.

[10] Jiu M., Pustelnik N. (2021). A deep primal-dual proximal network for image restoration. *IEEE Journal of Selected Topics in Signal Processing*.

[11] Agnes S. S., Akshaya D., Kaviya M., Kiruthiga K. (2020). A comprehensive survey on crack detection of bone using various techniques. *Bulletin of Scientific Research*.

[12] Zheng X. (2020). Rationality modeling of 3D scanning image of digital print laser based on block matching texture information repair. *IEEE Sensors Journal*.

[13] Neilson B. N., Craig C. M., Curiel R. Y., Klein M. I. (2021). Restoring attentional resources with nature: a replication study of Berto's (2005) paradigm including commentary from Dr. Rita Berto. *Human Factors: The Journal of Human Factors and Ergonomics Society*.

[14] Espriella M. C., Lecours V., Frederick P. C., Camp E. V., Wilkinson B. (2020). Quantifying intertidal habitat relative coverage in a Florida estuary using UAS imagery and GEOBIA. *Remote Sensing*.

[15] Song G., Wang H. (2021). Artificial intelligence-assisted fresco restoration with multiscale line drawing generation. *Complexity*.

[16] Salman N. H., Rafea S. (2020). The arithmetic coding and hybrid discrete wavelet and cosine transform approaches in image compression. *Xinan Jiaotong Daxue Xuebao/Journal of Southwest Jiaotong University*.

[17] Wang X., Wang H., Niu S. (2020). An intelligent forensics approach for detecting patch-based image inpainting. *Mathematical Problems in Engineering*.

[18] Sidorenko A. V., Shakinko I. V. (2020). The digital watermarking algorithm using discrete chaotic maps. *system analysis and applied information science*.

[19] Yatnalli V., Shivaleelavathi B. G., Sudha K. L. (2020). Review of inpainting algorithms for wireless communication application. *Engineering, Technology and Applied Science Research*.

[20] Wang S., Xia K., Wang L., Zhang J., Yang H. (2020). Improved RPCA method via non-convex regularisation for image denoising. *IET Signal Processing*.

[21] Molina J., Ponomaryov V., Reyes R., Sadovnychiy S., Cruz C. (2020). Watermarking framework for authentication and self-recovery of tampered colour images. *IEEE Latin America Transactions*.

[22] Fan J., Wang Z., Lin M., Fang S., Liu X., Fan B. (2020). Research on vehicle attitude and heading reference system based on multi-sensor information fusion. *Proceedings of the Institution of Mechanical Engineers, Part D: Journal of Automobile Engineering*.

[23] Liu Y., Hu W., Han L., Taras M., Chen Z. (2020). A fast filling algorithm for image restoration based on contour parity. *Computers, Materials and Continua*.

[24] Fan M., Sharma A. (2021). Design and implementation of construction cost prediction model based on SVM and LSSVM in industries 4.0. *International Journal of Intelligent Computing and Cybernetics*.

[25] Raj M., Manimegalai P., Ajay P., Amose J. (2021). Lipid data acquisition for devices treatment of coronary diseases health stuff on the Internet of Medical Things. *Journal of Physics: Conference Series*.

[26] Liu Q., Liu X., Liu T., Kang Y., Zhang H. (2020). Seasonal variation in particle contribution and aerosol types in Shanghai based on satellite data from MODIS and CALIOP. *Particuology*.

[27] Huang R., Zhang S., Zhang W., Yang X. (2021). Progress of zinc oxide-based nanocomposites in the textile industry. *IET Collaborative Intelligent Manufacturing*.

[28] Guo E., Jagota V., Makhatha M., Kumar P. (2021). Study on fault identification of mechanical dynamic nonlinear transmission system. *Nonlinear Engineering*.

